# Men with Latent Autoimmune Diabetes and Type 2 Diabetes May Have Different Change Patterns in Free Testosterone

**DOI:** 10.1155/2020/6259437

**Published:** 2020-07-24

**Authors:** Bo Ding, Feng-fei Li, Xiao-fang Zhai, Lei Ye, Yun Hu, Jian-hua Ma

**Affiliations:** ^1^Department of Endocrinology, Nanjing First Hospital, Nanjing Medical University, Nanjing, China; ^2^National Heart Research Institute Singapore, National Heart Centre Singapore, Singapore

## Abstract

**Objective:**

Type 2 diabetic (T2D) male patients with low total testosterone (TT) levels are at an increasing risk of all-cause mortality. However, the levels of TT in male patients with latent autoimmune diabetes in adults (LADA) remain largely unknown. *Research Design and Methods*. This was a single-center, open, observational study. The inclusion criteria were male patients who were diagnosed with LADA, and sex, body mass index, C-peptide, and glycated hemoglobin (HbA1c) levels matched with those of T2D patients. Islet function/sensitivity and sex hormone concentrations were determined at baseline and 1-year follow-up. The primary endpoint was the changes in androgen levels from baseline to 1-year follow-up in patients with LADA.

**Results:**

Our data showed that TT and Bio-T levels remained unchanged, while FT levels significantly decreased from baseline to 1-year follow-up in patients with T2D. However, TT, Bio-T, and FT concentrations dramatically increased in the LADA group from baseline to 1-year follow-up. Furthermore, a Spearman analysis showed that changes of TT, FT, and Bio-T levels from baseline to endpoint were significantly negatively correlated with *Δ* homeostasis model assessment-2 IR (*Δ*HOMA2-IR), respectively.

**Conclusions:**

The FT change patterns in patients with LADA may differ from those in patients with T2D. Our data also indicated the significant negative correlation between insulin sensitivity and changes of TT, FT, and Bio-T levels along with the diabetic duration in patients with T2D and LADA.

## 1. Introduction

Aging is a well-known risk factor for type 2 diabetes (T2D), causing a decrease in insulin production and sensitivity cells [1, 2]. Endogenous sex hormones decrease in men and women with age [1, 2], which differently modulate glycemic metabolism between the subjects [3]. Evidence indicates that testosterone concentrations are positively correlated to T2D in women but negatively associated in men; women who had high sex hormone-binding globulin (SHBG) levels also benefited more from reducing incidence of T2D than did men [3]. Researchers further observed that high total testosterone (TT) and free testosterone (FT) values have a potential protective role in reducing the risk of T2D in elderly men [4]. In agreement with this study, a prospective study found that low TT levels are associated with an increase in T2D in men [5], especially in obese T2D male patients with or without metabolic syndrome [6]. Moreover, T2D patients with low T levels had poor glycemic control and increased insulin resistance, which may contribute to the longer duration of diabetes [7]. Very recently, researchers confirmed that type 2 diabetic men, especially those with low TT concentrations, have increased all-cause mortality [8, 9], leading to a high prevalence of worsening cardiac function, ischemia, and readmission rate [8].

Few studies have focused on sex hormones in patients with type 1 diabetes (T1D). However, previous data suggest that sex hormone concentrations in men with T1D may not be the same as in those with T2D [10]. A previous study showed that the incidence of TT deficiency in male patients with T1D was similar to that in healthy men [11]. Furthermore, a study demonstrated that patients with T1D have higher levels of TT, FT, and SHBG than those in patients with T2D [12]. However, the increased androgen levels had no correlation with insulin sensitivity in T1D adolescents [13]. The underlying mechanisms may be the increased androgen synthesis [14] and the inhibitory effect of insulin on SHBG production in the liver [10].

Latent autoimmune diabetes in adults (LADA) is the most frequent form of autoimmune diabetes, with a higher prevalence than that of adult-onset T1D [15]. The term “type 1.5 diabetes” describes the clinical features of LADA: patients with LADA lack insulin dependency and positive islet autoantibodies at onset, but with a faster decline in beta cell function, they become insulin dependent during the duration progression [16]. Studies have already demonstrated that sex hormone concentrations differ between patients with T2D and T1D, which play a potential role in the risk of incidence and mortality in the two groups. However, research studies focusing on sex hormone change patterns in patients with LADA are mainly unclear.

Therefore, we performed a single-center, open, retrospective study. In this study, we compared the change in patterns of androgen concentrations between patients with LADA and T2D from baseline to 1-year follow-up.

## 2. Research Design and Methods

This was a single-center, open, observational study. The study protocol and patient consent forms were approved by the Institutional Ethics Committee of Nanjing First Hospital, Nanjing Medical University, No. 32, Gongqingtuan Road, Nanjing, China (2015KY07). All patients provided written informed consent to participate. The methods were conducted in accordance with the Declaration of Helsinki guidelines, including any relevant details.

The inclusion criteria were drug-naïve male patients who were diagnosed with LADA (*n* = 10) or T2D (*n* = 15) at Nanjing First Hospital by research clinicians. The criteria for diagnosis of LADA were proposed by the Chinese Diabetes Society: (1) the presence of any islet autoantibodies (glutamic acid decarboxylase antibody (GADA), and the combination of tyrosine phosphatase-like protein antibody (IA-2A), insulin autoantibody (IAA), and autoantibodies to zinc transporter 8 (ZnT8A), can increase the detection rate); (2) the onset age ≥ 18 years; and (3) a minimum period of 6 months of insulin independence. The exclusion criteria were as follows: (a) patients who used systemic steroidal anti-inflammatory drugs or any drugs that may influence T level in the last 3 months; (b) patients with an acute infection; (c) patients with acute complications of diabetes; and (d) patients with a severe systemic disease or any other condition that is judged by researchers to be unsuitable for this study. All enrolled patients were admitted to Nanjing First Hospital in China between March 2016 and January 2019, and the observation period was 12 months.

### 2.1. Clinical and Laboratory Assessments

Demographic data in terms of height, weight, and age were recorded at baseline and endpoint. Fasting serum was collected for glucose, glycated hemoglobin (HbA1c), C-peptide, albumin, lipid profiles, TT, and SHBG at baseline and 1-year follow-up, respectively. Bioavailable testosterone (Bio-T) and FT were calculated based on TT, SHBG, and albumin levels. A standard meal test was performed to measure glucose and C-peptide concentrations 120 min after meal loading. HbA1c was measured using a high-performance liquid chromatography assay (Bio-Rad Laboratories, Inc., Hercules, CA, USA). C-peptide was determined by chemiluminescent immunometric assay, which employs the Modular Analytics E170 (Roche Diagnostics GmbH, Mannheim, Germany). TT and SHBG were measured using a chemiluminescent immunometric assay, which employs a UniCel™ Dxl 800 automated analyzer (Beckman Coulter Inc., Brea, CA, USA). Body mass index (BMI) was calculated as weight divided by the square of height (kg/m^2^). Homeostasis model assessment-2 IR (HOMA2-IR) was calculated as previously described [17]. The inclusion criteria for T2D were age, sex, FBG, HbA1c, and fasting C-peptide (<0.75 ng/mL) [7], matched with LADA patients.

All patients enrolled in our study were treated with premixed insulin analog combination with metformin for a year, and the study design was described in the study flow chart (Figure 1).

### 2.2. Statistical Analysis

Statistical analysis was performed using SPSS 16.0 software (SPSS, Science, Chicago, IL, USA). All variables were tested for normal distribution of the data. Data are presented as the mean ± standard error (SE). A paired sample *t*-test was used for intragroup comparison, and an independent sample *t*-test was used for intergroup comparison. A Spearman analysis was employed to analyze the regression relationships. All comparisons were 2-sided at a 5% significance level. A *P* value of less than 0.05 was considered statistically significant.

## 3. Results

### 3.1. Demographic and Glucose-Lowering Agent Profiles of Enrolled Patients

From January 2016 to June 2019, 25 male patients with LADA (*n* = 10) and male patients with T2D (*n* = 15) were enrolled into this study, and all patients completed this study. The demographic characteristics are described in detail in Table 1. Patients with LADA had similar age, FBG, HbA1c, fasting C-peptide, TC, TG, HDL, and LDL concentrations at baseline compared with patients with T2D, and patients in the T2D group had a significant increase in postprandial C-peptide levels (Table 1). Patients with LADA and T2D need insulin (0.46 ± 0.07 IU/kg, 0.48 ± 0.05 IU/kg, respectively) and metformin (1285.71 ± 267.26 mg, 1285.71 ± 267.26 mg, respectively) to maintain glycemic control at the endpoint.

### 3.2. Changes in Islet Beta Cell Function and Insulin Sensitivity

Fasting and postprandial C-peptide levels in patients with LADA significantly decreased from baseline to 1-year follow-up. On the other hand, patients with T2D had significantly increased islet function. We also compared insulin sensitivity using the HOMA2-IR index between the two groups. We observed that the HOMA2-IR value significantly increased in patients with T2D from baseline to 1-year follow-up, while in patients with LADA, it remained unchanged (Table 2). Furthermore, our data indicated that patients with LADA had significant improvement in insulin sensitivity from baseline to 1-year follow-up, compared with patients in the T2D group (Table 3).

### 3.3. Changes in HbA1c and Sex Hormone Levels from Baseline to 1-Year Follow-Up

We further compared the changes in HbA1c and sex hormone levels between the two groups at the endpoint. We observed that the levels of TT, Bio-T, and FT values significantly increased in patients with LADA from baseline to 1-year follow-up. Contrary to the trend in the T2D group, patients with T2D had similar TT and Bio-T levels, with a significant decrease in FT value from baseline to endpoint. We also analyzed the changes in SHBG levels between the two groups from baseline to endpoint. Our data showed that SHBG levels were unchanged within the two groups; however, patients with LADA had higher SHBG levels than those of T2D patients at baseline and at the endpoint, respectively (Figure 2).

### 3.4. Factor(s) That Contributed to Changes in Sex Hormone Levels from Baseline to Endpoint

To identify which factor(s) that contributed to the changes in SHBG, TT, FT, and Bio-T in patients with diabetes, a Spearman analysis was performed. Our data showed that *Δ*TT, *Δ*FT, and *Δ*Bio-T levels were significantly positively correlated with GADA levels at baseline (all *P* < 0.05), while being significantly negatively correlated with changes in fasting and postprandial C-peptide concentrations from baseline to endpoint (all *P* < 0.05). We did not observe any correlation relationships regarding *Δ*SHBG levels with the abovementioned factors. Importantly, we observed a significant negative correlation between HOMA2-IR and *Δ*TT, *Δ*FT, and *Δ*Bio-T levels (*P* < 0.05) (Table 4).

## 4. Discussion

This relatively modest study revealed a novel observation that the FT level change pattern in male patients with LADA differed from age- and sex-matched patients with T2D, which gradually decreased along with the diabetic progression. Our data suggested that the change in insulin sensitivity may contribute to the different change patterns between patients with LADA and T2D. Our data also indicated a significant negative correlation between insulin sensitivity and changes of TT, FT, and Bio-T levels along with the diabetic duration in patients with T2D and LADA.

A systematic review and meta-analysis showed that high SHBG concentrations were associated with a high reduction in incidence of T2D in women (>60 nmol/L) compared with men (>28.3 nmol/L) [3]. In contrast, another study showed that women and men with low circulating SHBG concentrations had a high risk of T2D [18]. The cutoff points for men and women at a high risk for T2D might be SHBG values < 40 and <50 nmol/L, respectively [19]. In this study, we observed that patients with T2D had low SHBG levels (<50 nmol/L), while subjects with LADA had high SHBG values (>50 nmol/L), with no changes along with the 1-year follow-up in each group. However, we found that patients with LADA had significantly increased SHBG levels at onset and endpoint, and low SHBG levels may be a potential risk factor for glycemic control in patients with T2D, independent of both adiponectinemia and insulinemia [20]. We observed that male patients with LADA had significant worsening of fasting glucose control compared to males with T2D at the endpoint. The underlying mechanism for uncontrolled glycemia may be the deterioration of beta cell function and the increased insulin sensitivity in patients with LADA. Hence, future studies are needed to identify the role of SHBG in regulating glycemia in patients with LADA.

In humans, TT status consists of Bio-T and conjugated T, with SHBG and albumin as the two bounding proteins [21]. In serum, FT and T conjugated to albumin are called Bio-T [22]. T plays a potential role in controlling carbohydrate metabolism [23]. It also increases glucose uptake via the activation of glucose transporter (GLUT-4) in the liver, adipose tissue, and muscle [24, 25]. In addition, studies have shown that T increases glycolysis and glycogen synthesis and reduces glycogen decomposition of skeletal muscle partially, by enhancing phosphofructokinase and hexokinase [26, 27]. Moreover, T may directly ease the process of glucose stimulation insulin secretion via binding to androgen receptors on islet *β* cells [28]. Therefore, T plays an important role in regulating glucose control in patients with diabetes. In this study, we observed a difference in androgen change patterns in patients with LADA and T2D. The TT, FT, and Bio-T levels significantly increased in the LADA group, while FT levels significantly decreased in patients with T2D. Furthermore, changes in TT, FT, and Bio-T concentrations significantly increased in the LADA group from baseline to endpoint, while these change directions were opposite in T2D patients. However, the underlying mechanisms of the two different changing tendencies of androgen concentrations should be elucidated in future studies. This has been addressed as a limitation in the study.

It is unclear which of these forms of T status are the most appropriate ones regulating metabolism. Studies showed that TT should be considered an indicator of metabolic syndrome rather than other forms of T should [29]. Our data showed that patients with LADA and T2D had similar TT values at onset. However, we observed a significant increase in TT levels in the LADA group from onset to 1-year follow-up.

Androgens play an important role in both muscle mass and body fat remodeling, both of which are correlated with insulin resistance [23]. However, the relationships between variations in T levels and metabolic conditions remain unclear. A study indicated that the low T level in men was an independent risk factor for metabolic syndrome [30]. Furthermore, most obese T2D patients were found with low T levels [31, 32]. In this study, we observed that androgen levels, especially FT and Bio-T values, in the LADA group were significantly increased, while the body weight remained unchanged from onset to endpoint. This warrants the study identifying the relationship between androgen level and weight gain in subjects with LADA.

In conclusion, The FT change patterns in patients with LADA may differ from those in patients with T2D. Our data indicated that insulin sensitivity may contribute to the different FT change patterns in patients with T2D and LADA.

## Figures and Tables

**Figure 1:** The study flow chart.

**Figure 2:** Changes of sex hormones from baseline to 1-year follow-up between the two groups.

**Table 1:** Demographic characteristics and serum parameters between the two groups at baseline and after 1-year follow-up.

	Baseline			After 1 year		
Items	LADA	T2D	*P*	LADA	T2D	*P*
Age	52.6 ± 17.5	49.9 ± 10.2	0.63	53.6 ± 17.5	50.9 ± 10.2	0.64
BMI	22.2 ± 3.2	23.7 ± 2.6	0.23	22.1 ± 3.3	23.8 ± 2.3	0.26
Albumin	38.5 ± 3.3	40.9 ± 1.8^∗^	0.03	42.2 ± 4.2	44.1 ± 3.2	0.25
TC	4.7 ± 1.2	4.8 ± 0.7	0.85	4.3 ± 0.8	4.1 ± 0.4	0.51
TG	1.0 ± 0.5	1.6 ± 1.6	0.30	1.0 ± 0.7	1.2 ± 0.5	0.42
HDL-C	1.4 ± 0.4	1.2 ± 0.3	0.31	1.6 ± 0.5	1.4 ± 0.2	0.33
LDL-C	2.6 ± 0.7	2.2 ± 0.6	0.38	1.8 ± 0.5	1.7 ± 0.3	0.58

LADA: latent autoimmune diabetes in adults; BMI: body mass index (kg/m^2^); TC: total cholesterol (mmol/L); TG: total triglycerides (mmol/L); HDL-C: high-density lipoprotein cholesterol (mmol/L); LDL-C: low-density lipoprotein cholesterol (mmol/L).

**Table 2:** Islet function and insulin sensitivity between the two groups at baseline and after 1-year follow-up.

	Baseline			After 1 year		
Items	LADA	T2D	*P*	LADA	T2D	*P*
FBG	10.1 ± 4.4	8.5 ± 3.6	0.38	10.4 ± 4.3	7.5 ± 1.2	0.06
HbA1c	10.3 ± 2.6	9.3 ± 1.7	0.29	9.0 ± 2.5	8.1 ± 1.2	0.24
C-p0 min	0.5 ± 0.3	0.6 ± 0.2	0.14	0.2 ± 0.2	1.3 ± 0.8^∗^	0.001
C-p120 min	0.6 ± 0.5	2.0 ± 0.8^∗^	0.001	0.3 ± 0.3	4.2 ± 1.3^∗^	0.001
HOMA2-IR	7.3 ± 4.0	8.2 ± 4.0	0.65	3.7 ± 2.8	12.7 ± 6.4^∗^	0.001

LADA: latent autoimmune diabetes in adults; FBG: fasting blood glucose (mmol/L); C-p0 min: C-peptide 0 min (ng/mL); C-p120 min: C-peptide120 min (ng/mL); HOMA2-IR: homoeostasis model assessment-2 insulin resistance.

**Table 3:** Changes of A1c, sex hormone, and insulin sensitivity between the two groups (values of 1-year follow-up minus values of baseline).

Items	LADA group	T2D group	*P* values
*Δ*HbA1c	−1.2 ± 2.3	−1.4 ± 1.0	0.78
*Δ*TT	6.5 ± 4.3	−1.3 ± 3.9^∗^	0.001
*Δ*FT	0.1 ± 0.1	−0.0 ± 0.1^∗^	0.001
*Δ*Bio-T	2.9 ± 1.6	−0.5 ± 1.7^∗^	0.001
*Δ*SHBG	0.2 ± 9.5	0.1 ± 10.4	0.98
*Δ*HOMA2-IR	−4.9 ± 5.5	4.7 ± 6.5^∗^	0.01

*Δ*HbA1c: HbA1c (%); *Δ*TT: total testosterone (nmol/L); *Δ*FT: free testosterone (nmol/L); *Δ*Bio-T: bioavailable testosterone (nmol/L); *Δ*SHBG: sex hormone-binding globulin (nmol/L); *Δ*HOMA2-IR: HOMA2-IR: homoeostasis model assessment-2 insulin resistance.

**Table 4:** Factor(s) that contributed to changes of sex hormone levels from baseline to endpoint.

	GADA 1		*Δ*C-p0 min		*Δ*C-p120 min		*Δ*HOMA2-IR	
	*r*	*P*	*r*	*P*	*r*	*P*	*r*	*P*
*Δ*TT	0.72	0.001	-0.70	0.001	-0.73	0.01	-0.67	0.01
*Δ*FT	0.68	0.001	-0.64	0.001	-0.69	0.03	-0.70	0.01
*Δ*Bio-T	0.61	0.01	-0.65	0.001	-0.72	0.02	-0.65	0.01

GADA 1: glutamic acid decarboxylase antibody at baseline (IU/mL); *Δ*C-p0 min: C-peptide 0 min (value of 1-year follow-up) − C-peptide 0 min (value of baseline); *Δ*C-p 120 min: C-peptide 120 min (value of 1-year follow-up) − C-peptide 120 min (value of baseline); *Δ*TT: TT (value of 1-year follow-up)−TT (value of baseline); *Δ*FT: FT (value of 1-year follow-up)−FT (value of baseline); *Δ*Bio-T: Bio-T (value of 1-year follow-up)−Bio-T (value of baseline); *Δ*HOMA2-IR: HOMA2-IR (value of 1-year follow-up)−HOMA2-IR (value of baseline).

## Data Availability

The datasets generated during and/or analyzed during the current study are not publicly available due [REASON WHY DATA ARE NOT PUBLIC] but are available from the corresponding author on reasonable request.
